The article "Associations of systemic oxygen consumption with age and body temperature under general anesthesia: retrospective cohort study" was retracted in 2023. Reasons: errors in the data; errors in the results or conclusions.

# Associations of systemic oxygen consumption with age and body temperature under general anesthesia: retrospective cohort study

**DOI:** 10.1186/s12871-023-02182-1

**Published:** 2023-06-20

**Authors:** Satoshi Kimura, Kazuyoshi Shimizu, Hiroshi Morimatsu

**Affiliations:** Department of Anesthesiology and Resuscitology, Okayama University Hospital, 2-5-1, Shikata-Cho, Kita-Ku, Okayama, 700-8558 Japan

**Keywords:** Oxygen Consumption, Body Temperature, General Anesthesia

## Abstract

**Background:**

Body temperature (BT) is thought to have associations with oxygen consumption (VO_2_). However, there have been few studies in which the association between systemic VO_2_ and BT in humans was investigated in a wide range of BTs. The aims of this study were 1) to determine the association between VO_2_ and age and 2) to determine the association between VO_2_ and BT.

**Methods:**

This study was a retrospective study of patients who underwent surgery under general anesthesia at a tertiary teaching hospital. VO_2_ was measured by the Dräger Perseus A500 anesthesia workstation (Dräger Medical, Lubeck, Germany). The associations of VO_2_ with age and BT were examined using spline regression and multivariable regression analysis with a random effect.

**Results:**

A total of 7,567 cases were included in this study. A linear spline with one knot shows that VO_2_ was reduced by 2.1 ml/kg/min with one year of age (*p* < 0.001) among patients less than 18 years of age and that there was no significant change in VO_2_ among patients 18 years of age or older (estimate: 0.014 ml/kg/min, p = 0.08). VO_2_ in all bands of BT < 36.0 °C was not significantly different from VO_2_ in BT >  = 36 °C and < 36.5 °C. Multivariable linear regression analysis showed that compared with VO_2_ in BT >  = 36 °C and < 36.5 °C as a reference, VO_2_ levels were significantly higher by 0.57 ml/kg/min in BT >  = 36.5 °C and < 37 °C (*p* < 0.001), by 1.8 ml/kg/min in BT >  = 37 °C and < 37.5 °C (*p* < 0.001), by 3.6 ml/kg/min in BT >  = 37.5 °C and < 38 °C (*p* < 0.001), by 4.9 ml/kg/min in BT >  = 38 °C and < 38.5 °C (*p* < 0.001), and by 5.7 ml/kg/min in BT >  = 38.5 °C (*p* < 0.001). The associations between VO_2_ and BT were significantly different among categorized age groups (*p* = 0.03).

**Conclusions:**

VO_2_ increases in parallel with increase in body temperature in a hyperthermic state but remains constant in a hypothermic state. Neonates and infants, who have high VO_2_, may have a large systemic organ response in VO_2_ to change in BT.

**Supplementary Information:**

The online version contains supplementary material available at 10.1186/s12871-023-02182-1.

## Background

Oxygen consumption (VO_2_) is an important part of hemodynamic assessment in critically ill patients. Since inadequate oxygen delivery for VO_2_ has been shown to be related to a severe condition of the patient and poor outcomes, one of the main goals in the operating room and intensive care unit is to maintain the balance of systemic oxygen supply and VO_2_ [1–3]. Although efforts should be made to maintain adequate systemic oxygen delivery, such efforts are sometimes not sufficient for patients with cardiac dysfunction and patients in whom there is a negative hemodynamic impact of sedative and analgesic agents. In such situations, reduction of VO_2_ could be a reasonable option to balance oxygen supply–demand.

The article "Associations of systemic oxygen consumption with age and body temperature under general anesthesia: retrospective cohort study" was retracted in 2023. Reasons: errors in the data; errors in the results or conclusions.

Body temperature (BT) is thought to have associations with oxygen consumption. For example, hypothermia has been used as a treatment for postischemic neurological injury [4, 5]. One of the theories regarding the effectiveness of the therapeutic hypothermia is that cerebral metabolism and oxygen consumption decrease during cooling [5]. In fact, many studies have confirmed an association between cerebral oxygen consumption and BT [6–8]. Hypothermia during cardiopulmonary bypass is another example. Hypothermia during cardiopulmonary bypass is expected to be effective for protecting not only the brain but also other organs such as the kidneys [9–11]. Body temperature control has also been employed as a strategy for postoperative cardiac patients with refractory low cardiac output syndrome, especially in pediatric patients with a relatively high oxygen demand [12, 13]. However, there have been few studies on the association between systemic VO_2_ and BT in humans in a wide range of BTs: between mild to moderate hypothermia and hyperthermia.

There are various methods for measuring VO_2_. Indirect calorimetry has long been acknowledgement as a gold standard reference tool [14]. Mass spectroscopy also enables accurate measurements of VO_2_ [15]. However, those methods require special equipment that is cumbersome and costly and they are not used in daily clinical practice. As an alternative, Sykes proposed an equation for estimating VO_2_ using data obtained from an oxygen sensor installed in an anesthesia breathing circuit [16]. By measuring the inspired oxygen fraction, expired oxygen fraction, and minute ventilation and using the formula, recent anesthesia workstations can provide data for VO_2_ breath-by-breath and can also provide a large amount of data in daily clinical practice.

We hypothesized that systemic VO_2_ during anesthesia has a linear association with BT ranging from low BT to high BT in both adult and pediatric patients. The aims of this study were 1) to determine the association of VO_2_ based on Sykes’ formula with age and 2) to determine the association of VO_2_ with BT.

The article "Associations of systemic oxygen consumption with age and body temperature under general anesthesia: retrospective cohort study" was retracted in 2023. Reasons: errors in the data; errors in the results or conclusions.

## Methods

### Design, study population and management

This study was a retrospective study of patients who underwent surgery under general anesthesia at a tertiary teaching hospital (Okayama University Hospital, Japan) during the period from May 2018 to October 2022. Patients with data for VO_2_ during surgery were included in this study. Patients without data for core body temperature, patients who underwent surgery with cardiopulmonary bypass, patients who underwent a second or subsequent surgery, and patients who were managed with an uncuffed endotracheal tube were excluded from this study.

BT was monitored at the nasopharynx, deep forehead, urinary bladder, or rectum during anesthesia. The site of BT monitoring, the use of forced-air cutaneous cover blankets and target BT during anesthesia were dependent on anesthesiologists who were responsible for each patient. The study was approved by the Okayama University Hospital Ethics Committee (Institutional Review Board Approval Number 2301–034), and the need for informed consent was waived. All regulations and measures of ethics and confidentiality were handled in accordance with the Declaration of Helsinki.

### Study variables and data sources

Patients’ information was stored in a central server and subsequently exported for further analyses through a medical data recording system, Prescient CDM (FUJIFILM Medical IT Solutions Co., Ltd., Tokyo, Japan), and additional information was obtained from electronic patient medical records.

VO_2_ was measured by the Dräger Perseus A500 anesthesia workstation (Dräger Medical, Lubeck, Germany) using Sykes’ formula [16]: VO_2_ = (FiO_2_—ETO_2_) × MV, where FiO_2_ is the inspired oxygen fraction, ETO_2_ is the expired oxygen fraction and MV is minute ventilation. VO_2_ was recorded minute-by-minute in the CDM system. BT during anesthesia was also recorded minute-by-minute in the CDM system. In cases with multiple monitors for core body temperature, the mean of the measurements was used for analysis. Data on VO_2_ and BT between the beginning of surgery and the end of surgery were extracted from the CDM system.

### Statistical analysis

Data are presented as frequency and proportion or median (IQR, interquartile range; 25% quartile to 75% quartile) as appropriate. For groupwise comparisons of continuous variables, the Wilcoxon rank sum test (two groups) or Kruskal–Wallis test (more than two groups) was used. For categorical variables, Fisher’s exact test or the chi-square test was used as appropriate.

First, the association between age and VO_2_ measured in this study was assessed. Data for VO_2_ when BT was between 36 degrees Celsius (°C) and 36.5 °C as normothermia were used and the mean of VO_2_ in each patient was used for analysis to make the assumption that observations were independent. The correlations between VO_2_ and age were assessed by Pearson’s correlation coefficients with 95% confidence interval (CI). A scatter plot was shown, and assuming that the relationship would be different in pediatrics and adults, a cubic spline and a linear spline with one knot (18 years of age) were used. Patients were also classified by age categories: (A) < 1 year of age, (B) >  = 1 year of age and < 5 years of age, (C) >  = 5 years of age and < 18 years of age, and (D) >  = 18 years of age. In order to better assess the association between VO_2_ and age in young pediatric patients using cubic spline regression, subgroup analysis for the association in patients less than 5 years of age was also conducted.

The article "Associations of systemic oxygen consumption with age and body temperature under general anesthesia: retrospective cohort study" was retracted in 2023. Reasons: errors in the data; errors in the results or conclusions.

Second, the association between VO_2_ measured in this study and BT was assessed. All data for VO_2_ were used for the analysis. Since the relationship between body temperature and VO_2_ might not be linear, BT was stratified into bands of 0.5 °C in width and handled as a categorical variable. The mean of VO_2_ in every range of BT was calculated for each patient, and data distribution in each range of BT was shown using box plots. VO_2_ in each BT category was compared with VO_2_ in BT of 36 °C and 36.5 °C as a reference using univariate regression analyses.

A linear mixed effects model was also used to assess the association between VO_2_ and BT, accounting for within-subject correlations resulting from the repeated measures. In the model, random intercept was assumed to capture potential differences in the references among individuals, with the covariance structure of compound symmetry. Categorized age, categorized BT and gender were included in the model. Since there was a possibility that there would be difference in the association between VO_2_ and BT depending on the age of the patient, subgroup analyses were performed in categorized age groups. Repeated-measures analysis of variance test was used to assess the differences in the associations between VO_2_ and BT among categorized age groups.

With use of a paired t-test, a sample size of 128 provided an 80% power, at a 0.05 two-sided significance level, to detect a mean of the differences of 0.05 ml/kg/min with a standard deviation of 0.2 ml/kg/min between two BT categories. A complete case analysis for each analysis was performed. All statistical comparisons were two-sided and a significance level was defined as a *P* value of less than 0.05. All statistical analyses were performed using R 3.6.0 (R Foundation for Statistical Computing, Vienna, Austria).

The article "Associations of systemic oxygen consumption with age and body temperature under general anesthesia: retrospective cohort study" was retracted in 2023. Reasons: errors in the data; errors in the results or conclusions.

## Results

### Participants

A total of 11,066 cases were considered to be eligible in the study. After excluding 3,499 cases according to the exclusion criteria, 7,567 patients were included in this study (Fig. 1). The demographic parameters in the primary cohort are shown in Table 1. Out of all patients, 131 (1.7%) were younger than one year, 192 (2.5%) were between one and five years old, 552 (7.3%) were between five and 18 years old, and 6,692 (88.4%) were 18 years old or older. The median number of VO_2_ measurements was 151 (IQR 84 to 251) per patient.

**Fig. 1:** Flow chart

**Table 1:** Demographics parameters

Variable	*n* = 7,567
Age, years [IQR]	61.00 [41.00, 72.00]
Weight, kg [IQR]	57.10 [48.20, 66.90]
Male, n (%)	3560 (47.0)
Duration of anesthesia, (hours) [IQR]	3.83 [2.52, 5.67]
Duration of surgery, (hours) [IQR]	2.63 [1.50, 4.30]

*Abbreviations*: *IQR* interquartile range

### Oxygen consumption among all ages

Figure 2 shows scatter plots of VO_2_ and age under the condition of BT between 36 °C and 36.5 °C (*n* = 5,123) with a cubic spline and a linear spline with one knot (18 years of age). The Pearson correlation coefficient of VO_2_ vs. age was -0.29 (95% CI: -0.32 to -0.27, *p* < 0.001). The linear spline with one knot shows that VO_2_ was reduced by 2.1 ml/kg/min with one year of age (*p* < 0.001) among patients less than 18 years of age and that there was no significant change in VO_2_ among patients 18 years of age or older (estimate: 0.014 ml/kg/min, *p* = 0.08).

**Fig. 2:** Association between oxygen consumption and age with body temperature between 36 °C and 36.5 °C. Cubic spline (left) and linear spline with one knot at the age of 18 years (right) were drawn on the scatter plot of VO_2_ and age. Abbreviations: VO_2_, oxygen consumption

The results of multivariable linear regression analysis with a random effect are shown in Table 2. Compared with VO_2_ in patients >  = 18 years of age as a reference, VO_2_ levels were significantly higher by 35.3 ml/kg/min in patients < 1 year of age (*p* < 0.001), by 42.6 ml/kg/min in patients 1–5 years of age (*p* < 0.001), and by 14.4 ml/kg/min in patients 5–18 years of age (*p* < 0.001).

**Table 2:** Coefficients and estimates of the linear mixed effects model for oxygen consumption

	Estimate	se	*p*-value
Body temperature reference (36–36.5 °C)			
< 33 °C	-0.18	0.24	0.45
33–33.5 °C	-0.29	0.27	0.28
33.5–34 °C	-0.44	0.24	0.07
34–34.5 °C	0.34	0.23	0.15
34.5–35 °C	0.10	0.21	0.66
35–35.5 °C	-0.19	0.17	0.26
35.5–36 °C	-0.13	0.13	0.33
36.5–37 °C	0.57	0.11	< 0.001
37–37.5 °C	1.8	0.14	< 0.001
37.5–38 °C	3.6	0.21	< 0.001
38–38.5 °C	4.9	0.35	< 0.001
> = 38.5 °C	5.7	0.59	< 0.001
Male (vs. female)	1.8	0.23	< 0.001
Age reference (> = 18 years of age)			
< 1 year of age	35.3	0.87	< 0.001
1–5 years of age	42.6	0.72	< 0.001
5–18 years of age	14.4	0.44	< 0.001

*Abbreviations*: *se* standard error

The article "Associations of systemic oxygen consumption with age and body temperature under general anesthesia: retrospective cohort study" was retracted in 2023. Reasons: errors in the data; errors in the results or conclusions.

### Association between body temperature and systemic oxygen consumption

Figure 3 shows box plots of VO_2_ and sample sizes with data among BT bands of 0.5 °C in width. Compared with VO_2_ in BT >  = 36 °C and < 36.5 °C as a reference [41.3 (IQR 36.2 to 47.6) ml/kg/min], VO_2_ levels were significantly higher in BT >  = 36.5 °C and < 37 °C [41.9 (IQR 36.7 to 48.7) ml/kg/min, *p* < 0.001], BT >  = 37 °C and < 37.5 °C [44.3 (IQR 38.1 to 53.5) ml/kg/min, *p* < 0.001], BT >  = 37.5 °C and < 38 °C [48.9 (IQR 40.6 to 62.6) ml/kg/min, *p* < 0.001], BT >  = 38 °C and < 38.5 °C [56.2 (IQR 44.2 to 79.7) ml/kg/min, *p* < 0.001], and BT >  = 38.5 [59.3 (IQR 45.9 to 92.3) ml/kg/min, *p* < 0.001]. VO_2_ in all bands of BT < 36.0 °C was not significantly different from VO_2_ in BT >  = 36 °C and < 36.5 °C.

**Fig. 3:** Association between oxygen consumption and body temperature. Abbreviations: VO_2_, oxygen consumption; Ref, reference; *, *p* < 0.05; **, *p* < 0.01; *** *p* < 0.001

The result of the linear mixed effects model is shown in Table 2. Compared with VO_2_ in BT >  = 36 °C and < 36.5 °C as a reference, VO_2_ levels were significantly higher by 0.57 ml/kg/min in BT >  = 36.5 °C and < 37 °C (*p* < 0.001), by 1.8 ml/kg/min in BT >  = 37 °C and < 37.5 °C (*p* < 0.001), by 3.6 ml/kg/min in BT >  = 37.5 °C and < 38 °C (*p* < 0.001), by 4.9 ml/kg/min in BT >  = 38 °C and < 38.5 °C (*p* < 0.001), and by 5.7 ml/kg/min in BT >  = 38.5 °C (*p* < 0.001).

### Subgroup analyses for associations between body temperature and systemic oxygen consumption among categorized age groups

Results of subgroup analyses for the associations between VO_2_ measured and BT are shown in Supplemental Fig. S1, Supplemental Fig. S2, Supplemental Fig. S3, and Supplemental Fig. S4, respectively. In patients younger than one year old, compared with VO_2_ in BT >  = 36 °C and < 36.5 °C as a reference, VO_2_ levels were significantly higher in BT >  = 37.5 °C and < 38 °C, BT >  = 38 °C and < 38.5 °C, and BT >  = 38.5. In patients between one and five years old and patients between five and 18 years old, compared with VO_2_ in BT >  = 36 °C and < 36.5 °C as a reference, VO_2_ levels were significantly higher in BT >  = 37 °C and < 37.5 °C, BT >  = 37.5 °C and < 38 °C, BT >  = 38 °C and < 38.5 °C, and BT >  = 38.5. In patients 18 years old or older, compared with VO_2_ in BT >  = 36 °C and < 36.5 °C as a reference, VO_2_ levels were significantly higher in BT >  = 36.5 °C and < 37 °C, BT >  = 37 °C and < 37.5 °C, BT >  = 37.5 °C and < 38 °C, BT >  = 38 °C and < 38.5 °C, and BT >  = 38.5. The associations between VO_2_ and BT were significantly different among the groups (*p* = 0.03). The results of the linear mixed effects models in the subgroups are shown in Supplemental Table S1.

The article "Associations of systemic oxygen consumption with age and body temperature under general anesthesia: retrospective cohort study" was retracted in 2023. Reasons: errors in the data; errors in the results or conclusions.

## Discussion

In this retrospective study, we found that there was a significant reduction in VO_2_ with advance of age among patients less than 18 years of age but that there was no association between VO_2_ and age among patients 18 years of age or older. VO_2_ increased in parallel with increase in BT when BT was above 36.5 °C, but there was no significant change in VO_2_ when BT was below 36 °C. However, there were significant differences in the association between VO_2_ and BT among categorized age groups.

We found that VO_2_ was relatively stable and that there was no significant association between VO_2_ and age under the condition of normothermia in patients >  = 18 years of age. Linear mixed effects models with adjustment for body temperature also showed significantly higher VO_2_ in patients < 1 year of age, patients >  = 1 year of age and < 5 years of age, and patients >  = 5 years of age and < 18 years of age than that in patients >  = 18 years of age. The results showing high VO_2_ in children in this study are consistent with the results of previous studies [13, 17]. However, when discussing absolute measurements of VO_2_, especially among pediatrics, we have a concern about the reliability of measurements. VO_2_ measurements based on Sykes’ formula might be affected by the percentage of dead space and the levels of precision of flowmeters and ventilators [18, 19]. Errors arising from those concerns, especially in reading absolute numbers, would be an issue for small children.

The association between VO_2_ and BT is an issue of main interest in this study. There have been only a few studies in which the association between VO_2_ and temperature as a continuous variable or finely categorized variable was assessed, and the results were conflicting. Bacher et al. conducted a prospective study including 19 adult patients who underwent intracranial surgery and found that VO_2_ showed a trend for continuous decline with decrease in body temperature from 35.5 °C to 32.0 °C in a hypothermic group [20]. Holzinger et al. performed a prospective observational cohort study in 25 patients after cardiac arrest and reported continuous changes in VO_2_ between BTs of 33 °C and 37.6 °C, but they did not perform statistical analysis of the changes in VO_2_ [21]. Li et al. assessed VO_2_ after cardiopulmonary bypass in 20 children with congenital heart disease. In their observational study, the peak increase in VO_2_ was significantly correlated with the peak increase in central temperature between 36.6 °C and 38.4 °C [22]. Tokutomi et al. carried out a study in 31 patients with severe head injury to assess the effect of hypothermia on hemodynamics and metabolism. The results of their retrospective study showed that VO_2_ progressively decreased with hypothermia but showed smaller changes below 35 °C with no significant difference among the groups at BT below 35 °C [23]. Our results showing an association of VO_2_ with hyperthermia but not with hypothermia are consistent with the results of the studies by Tokutomi et al. and Li et al.[22, 23].

The article "Associations of systemic oxygen consumption with age and body temperature under general anesthesia: retrospective cohort study" was retracted in 2023. Reasons: errors in the data; errors in the results or conclusions.

Our study is the first study to show an association between VO_2_ and BT using a large number of subjects and our results suggested that hyperthermia increases VO_2_, but hypothermia does not reduce VO_2_. There are some explanations for our findings. First, hyperthermia increases VO_2_, but hypothermia below normal body temperature does not further decrease VO_2_ by systemic organs among patients under general anesthesia. All patients who underwent general anesthesia, not only patients with brain injury, were eligible for this study. Since sedation and neuromuscular blockade reduce VO_2_, VO_2_ in the patients in our study was considered to have been significantly suppressed [24–26]. A prospective observational study showed that VO_2_ decreased by a third after induction of anesthesia in elderly patients [27]. Further reduction in VO_2_ might not be possible in patients under general anesthesia. Second, there might be a confounding effect of anesthetic agents on the association between VO_2_ and BT. The effects of sedative agents and neuromuscular blocking agents on VO_2_ could not be separated appropriately due to the lack of data in our study and the magnitudes of their effects on VO_2_ under general anesthesia are still uncertain [24, 28]. Thus, there is a possibility that depression of hypothermia-induced cerebral electrical activity might need less doses of anesthetic agents, which offset the reduction in VO_2_ by hypothermia in this study [29].

Although our subgroup analyses among categorized age groups showed a significant difference in VO_2_ between hyperthermia and normothermia but no significant difference in VO_2_ between hypothermia and normothermia in all categorized age groups, there was a significant difference in the association between VO_2_ and BT among the groups. Here, the differences in VO_2_ among different BT categories in pediatric patients, especially patients less than 1 year of age, deserve separate mentioning. Being different from the trend of VO_2_ in other age groups, the absolute change in VO_2_ for the change in BT was large and the relationship between VO_2_ and BT was close to linear in the whole range of BTs among patients less than 1 year of age. These findings suggest that neonates and infants, who have high VO_2_ as shown in previous studies and in our study, might have a large systemic organ response in VO_2_ to change in BT and have the possibility for further reduction in VO_2_ even at BT below normal BT [13, 22]. No statistical significance in VO_2_ below normal BT might be due to small sample size and lack of power.

The article "Associations of systemic oxygen consumption with age and body temperature under general anesthesia: retrospective cohort study" was retracted in 2023. Reasons: errors in the data; errors in the results or conclusions.

Many strategies related to BT have been applied for patients with the belief that lower BT would decrease VO_2_ and protect systemic organs under the condition of inadequate oxygen delivery. For instance, hypothermia has been used to protect other organs such as the kidneys during cardiopulmonary bypass [9–11]. However, clinical studies have failed to show the superiority of deep hypothermia for prevention of acute kidney injury after cardiac surgery [30–32]. Our findings might provide an explanation for those results and our findings suggest that hyperthermia should be avoided for patients with limited oxygen delivery and that hypothermia might not reduce VO_2_ for protecting organs. However, our results suggesting that VO_2_ is not reduced by hypothermia in adult patients might not be applicable to pediatric patients.

There are several limitations in this study. First, the accuracy and precision of the VO_2_ measurements are issues. We used VO_2_ measurements based on Sykes’ formula, which might be affected by the percentage of dead space [18] and the levels of precision of flowmeters and ventilators [18, 19]. If the tidal volume (and thus the percentage of dead space) is unchanged, however, VO_2_ measurement using Sykes’ formula is a good indicator of whether VO_2_ is rising or falling [18]. Recording VO_2_ minute-by-minute and calculating the mean of VO_2_ in every range of BTs in each patient in this study would also have contributed to improvement in precision due to variance of the monitoring system. Thus, our assessment of VO_2_ compared with BT, especially the relative trend in VO_2_ with change in BT, would be acceptable. Second, the association between VO_2_ and BT would not indicate robust causal inference. We performed linear mixed effects models with adjustment for age and gender, and the results showed a significant association between VO_2_ and BT. However, since it is known that general anesthesia with sedation and neuromuscular blockade decrease VO_2_ and that thermoregulation is impaired during general anesthesia, anesthetic agents and the level of anesthesia might confound the association [24–26, 33]. The lack of those data in this study and the still uncertain effect of general anesthesia on VO_2_ makes it difficult to estimate the effect of BT on VO_2_ [24, 28]. Third, pulmonary artery temperature is considered the most accurate estimate of core temperature, whereas the BT measurements used in this study may be unreliable for estimating core body temperature. For example, bladder and rectal temperatures are less reliable due to poor perfusion and slower response during rapid changes in BT [34]. We excluded patients who underwent surgery with cardiopulmonary bypass, as they may require rapid temperature control. Additionally, in cases with multiple monitors, we calculated the average of the measurements to avoid relying on a potentially unreliable single measurement. However, a prospective study that monitors a single reliable location for body temperature would provide better assessment of the association between VO_2_ and BT.

The article "Associations of systemic oxygen consumption with age and body temperature under general anesthesia: retrospective cohort study" was retracted in 2023. Reasons: errors in the data; errors in the results or conclusions.

## Conclusions

VO_2_ increases in parallel with increase in body temperature in a hyperthermic state but remains constant in a hypothermic state. Neonates and infants, who have high VO_2_, might have a large systemic organ response in VO_2_ to change in BT and have the possibility for further reduction in VO_2_ even at BT below normal BT.

## Supplementary Information

**Additional file 1:  Figure S1.** Association between oxygen consumption and body temperature in patients younger than one year old. Abbreviations:VO_2_, oxygenconsumption; Ref, reference; *, *p*< 0.05; **, *p*< 0.01; *** *p*< 0.001

**Additional file 2: Figure S2.** Association between oxygen consumption and body temperature inpatients between one and fiveyears old. Abbreviations: VO_2_,oxygen consumption; Ref, reference; *, *p*< 0.05; **, *p*< 0.01; *** *p*< 0.001

**Additional file 3: Figure S3.** Association between oxygen consumption and body temperature inpatients between five and 18years old. Abbreviations: VO_2_,oxygen consumption; Ref, reference; *, *p*< 0.05; **, *p*< 0.01; *** *p*< 0.001

**Additional file 4: Figure S4.** Association between oxygen consumption and body temperature inpatients 18 years old or older. Abbreviations:VO_2_, oxygenconsumption; Ref, reference; *, *p*< 0.05; **, *p*< 0.01; *** *p*< 0.001

**Additional file 5: Table S1.**

## Data Availability

The datasets used and/or analyzed during the current study are available from the corresponding author on reasonable request.

## Abbreviations

VO_2_: Oxygen consumption
BT: Body temperature
FiO_2_: Inspired oxygen fraction
ETO_2_: Expired oxygen fraction
MV: Minute ventilation
IQR: Interquartile range
°C: Celsius
CI: Confidence interval
